# XRCC1 and hOGG1 polymorphisms and endometrial carcinoma: A meta-analysis

**DOI:** 10.1515/med-2024-0913

**Published:** 2024-03-04

**Authors:** Shengke He, Xiujuan Zhao, Ruifang Mu, Zhongjun Pan, Jinglan Mai

**Affiliations:** Department of Pathology, Danzhou People’s Hospital, Nada Town, Danzhou, Hainan, 571799, China; Department of Gynaecology and Obstetrics, Danzhou People’s Hospital, Nada Town, Danzhou, Hainan, 571799, China; Occupational Physical Examination Outpatient, Haikou Center for Disease Control and Prevention, No. 56 Yehai Avenue, Qiongshan District, Haikou, Hainan, 570203, China

**Keywords:** XRCC1-Arg399Gln, hOGG1-Ser326Cys, endometrial carcinoma, polymorphism, meta-analysis, genetic susceptibility

## Abstract

Endometrial carcinoma’s (EC) etiology is complex and involves DNA repair gene polymorphisms like XRCC1-Arg399Gln and hOGG1-Ser326Cys, but their association with the disease is unclear. Following PRISMA, we conducted a systematic review and meta-analysis, collecting data from four databases. The studies needed to be population-based case–control studies examining the association between the named polymorphisms and EC. Quality was assessed with the Newcastle-Ottawa Scale. Pooled odds ratios (OR) and 95% confidence intervals (CI) were calculated, and subgroup analyses were conducted based on ethnicity. Seven studies were included. Both polymorphisms were found to significantly increase EC risk, particularly in Caucasians. XRCC1-Arg399Gln showed a dominant model OR of 1.14 (95% CI: 1.01–1.29) and a homozygous model OR of 1.59 (95% CI: 1.12–2.25). The heterozygote model OR for hOGG1-Ser326Cys was 1.29 (95% CI: 1.02–1.63), and the allele OR was 1.31 (95% CI: 1.07–1.60). XRCC1-Arg399Gln and hOGG1-Ser326Cys may increase EC risk, primarily in Caucasian women, emphasizing the role of DNA repair in disease susceptibility. More extensive studies are needed to validate these findings in diverse ethnicities and investigate other DNA repair gene polymorphisms.

## 1 Introduction

Endometrial carcinoma (EC) is a heterogenous disease characterized by a group of epithelial malignant tumors localized in the uterine endometrium, the inner lining of the uterus. This neoplasia has drawn increasing global attention due to its rising incidence over the past several decades, with recent evidence indicating a clear upward trajectory across multiple geographical regions [1,2]. This trend is especially pronounced in developed countries like those in North America and Europe, where EC has surpassed other malignancies to become the most common gynecological cancer [3–5]. The etiology and pathogenesis of EC are multifactorial, with an array of both genetic and environmental risk factors implicated. An important constellation of metabolic disorders – obesity, hypertension, and diabetes, are often associated with EC. These conditions collectively underline the role of metabolic dysregulation in the pathogenesis of this malignancy [6–9]. DNA lesions arise due to a confluence of physiological/metabolic and external environmental variables. If left unaddressed, these modifications gradually accumulate within the cells as well as can lead to genetic mutations that alter the functionality of crucial proteins, such as tumor suppressors and oncoproteins. Additionally, they can cause rearrangements in the chromosomes, such as gene fusions, which further disrupt the regulation of essential cellular molecules [10–12].

The human body possesses an intricate DNA repair mechanism, an essential component of maintaining genomic stability [13,14]. This mechanism mitigates the potential harm resulting from DNA damage, preserving the integrity of the genome [15,16]. However, anomalies such as mutations or deletions in the DNA repair system can lead to genomic instability, setting the stage for oncogenic transformation [17]. Particular emphasis has been placed on two pivotal genes involved in the base excision repair (BER) pathway of the DNA repair system: X-ray repair cross-complementing gene 1 (XRCC1) and human 8-oxoguanine DNA glycosylase (hOGG1). Several studies have been investigating the potential associations of polymorphisms at specific loci of these genes, namely XRCC1 Arg399Gln and hOGG1 Ser326Cys, with EC susceptibility [18].

Previous research on the association of XRCC1-Arg399Gln and hOGG1-Ser326Cys polymorphisms with EC risk has yielded mixed results. For instance, studies such as those by Zhang and Li [19] and Romanowicz-Makowska et al. [20] have explored the relationship between XRCC1 Arg399Gln polymorphism and the risk of EC. Zhang and colleagues found a significant association between XRCC1 Arg399Gln and the susceptibility to gynecologic cancers, particularly cervical and endometrial cancers. In contrast, Romanowicz-Makowska et al. did not observe a significant association between XRCC1 Arg399Gln and different grades of endometrial cancer, although they noted a greater frequency of the XRCC1 399Gln allele in endometrial cancer patients. This suggests that while there might be a relationship with specific cancer subtypes, the association with endometrial cancer remains uncertain. Similarly, for the hOGG1 Ser326Cys polymorphism, studies by Shi et al. [21] and Krupa et al. [22] offer contrasting findings. Shi and colleagues reported a significant association between the hOGG1 Ser326Cys polymorphism and overall gynecologic cancer susceptibility, especially for endometrial cancer in the European population. On the other hand, Krupa et al. found no correlation between the Ser326Cys polymorphism of the hOGG1 gene and endometrial cancer. These conflicting results underscore the complexity of the genetic factors influencing EC and the need for further research in diverse populations. Through our systematic review and meta-analysis, we aim to reconcile the existing contradictions and provide a more comprehensive and definitive understanding of the role of XRCC1-Arg399Gln and hOGG1-Ser326Cys polymorphisms in the susceptibility to EC. This study is focused on assessing the associations between these polymorphisms and EC, taking into account various factors such as ethnicity, study design, and sample size, which are crucial in influencing the outcomes. By synthesizing diverse study results, our review endeavors to offer a nuanced understanding of how these genetic variations contribute to the development of EC. Moreover, the insights gained from this analysis are expected to have significant implications for personalized risk assessment, early detection strategies, and the development of targeted therapeutic interventions for EC.

## 2 Materials and methods

### 2.1 Search strategy

Throughout the systematic review procedure and subsequent presentation of our findings, we upheld compliance with the Preferred Reporting Items for Systematic Reviews and Meta-Analyses (PRISMA) guidelines [23]. On May 6, 2023, a search was conducted on four electronic databases, namely PubMed, Embase, Web of Science, and Cochrane Library. No temporal restrictions were imposed during the search. The specific search terms of PubMed were (“XRCC1” [All Fields] OR “X-ray repair cross-complementing gene 1” [All Fields] OR “Arg399Gln” [All Fields]) AND (“hOGG1” [All Fields] OR “human 8-oxoguanine DNA glycosylase” [All Fields] OR “Ser326Cys” [All Fields]) AND (“Endometrial Carcinoma” [MeSH Terms] OR (“Endometrial” [All Fields] AND “Carcinoma” [All Fields]) OR “Endometrial Carcinoma” [All Fields] OR (“Endometrial” [All Fields] AND “Cancer” [All Fields]) OR “Endometrial Cancer” [All Fields]) AND (“polymorphism, genetic” [MeSH Terms] OR (“polymorphism” [All Fields] AND “genetic” [All Fields]) OR “genetic polymorphism” [All Fields] OR “polymorphism” [All Fields]). No language limitation was applied. Reference lists of relevant articles were also screened manually for any additional possible records.

### 2.2 Inclusion criteria and exclusion criteria

Studies included in the systematic review needed to meet the following criteria: (1) Studies investigating the association between XRCC1 gene Arg399Gln polymorphism or hOGG1 gene Ser326Cys polymorphism and the risk of EC. (2) The study design must be a population-based case–control study. (3) The publication should provide the genotype frequencies for the test and control groups, enabling the calculation of odds ratios (OR) and their corresponding 95% confidence intervals (CI). (4) In the case of multiple publications from the same study, only the publication with the most comprehensive results will be included.

The exclusion criteria were as follows: (1) Reviews, abstracts, studies of poor quality, and studies for which valid data cannot be obtained after contacting the authors. (2) Studies not adhering to the case–control design. (3) Studies that do not meet the Hardy-Weinberg equilibrium (HWE) genetic balance.

### 2.3 Data extraction

The process of literature screening and data extraction will be conducted by two independent evaluators and subsequently cross-checked. In case of any inconsistencies encountered during this procedure, the reviewers involved are advised to engage in a discussion aimed at resolving the matter. If deemed necessary, a third reviewer may be consulted for further input. The data to be extracted included: first author’s name, year of publication, country where the study was conducted, sample size for both case and control groups, source of case and control groups, ethnicity of the study population, distribution frequency of various genotypes and alleles. In instances where the published report lacks pertinent data, communication is established with the original study’s investigators through electronic mail in order to solicit the unreleased data.

### 2.4 Quality assessment

The assessment of the studies incorporated in our meta-analysis will undergo a thorough evaluation by two autonomous reviewers utilizing the Newcastle-Ottawa Scale (NOS) to ensure their quality [24]. The NOS is a widely recognized instrument that assesses research studies according to nine distinct elements distributed across three fundamental domains, namely: selection, comparability, and outcome. The utilization of these categories facilitates the evaluation of potential sources of bias that may be inherent in the conducted studies. After conducting a thorough assessment, a numerical rating between 0 and 9 is allocated to each study to indicate its level of quality. The scoring system for the assessment of studies is as follows: studies that receive a score ranging from 0 to 3 are classified as low-quality research, those that score between 4 and 6 are considered to be of moderate quality, and those that achieve a score from 7 to 9 are categorized as high-quality research.

### 2.5 Statistical analyses

Heterogeneity among the studies will be assessed using the *Q*-test and *I* ^2^ statistic. If the *P*-value is greater than 0.10 or the *I* ^2^ statistic is less than 50%, indicating low heterogeneity, a fixed-effects model will be applied to calculate the pooled OR. In contrast, if there is significant heterogeneity (*P* ≤ 0.10 or *I* ^2^ ≥ 50%), a random-effects model will be used. Quantitative synthesis of the ORs and their 95% CI from the included studies will be carried out. The statistical significance of the pooled OR will be determined by the *Z*-test, with a *P*-value of less than 0.05 considered statistically significant. Forest plots will be created to graphically represent the results of the meta-analysis. Subgroup analyses will be performed based on ethnic variations in the study populations to explore potential sources of heterogeneity. The value of a two-sided *P* < 0.05 was considered statistically significant in all statistical tests. All statistical analyses will be conducted using Stata version 17 (StataCorp, College Station, TX, USA).

## 3 Results

### 3.1 Search results and study selection

Upon conducting an initial search of electronic databases, a total of 825 relevant literature sources were identified. Following the elimination of redundant literature, careful examination of titles and abstracts, and rigorous adherence to the established inclusion and exclusion criteria, a total of 20 relevant sources were identified, while 13 were deemed unsuitable for further analysis. Ultimately, a total of seven articles were included [18,22,25–29]. Figure 1 illustrates the process and outcomes of the literature screening.

**Figure 1:** Selection process of included studies.

### 3.2 Study characteristics

Our meta-analysis included studies that explored the polymorphisms of XRCC1 Arg399Gln and hOGG1 Ser326Cys in relation to EC. A total of six studies focused on XRCC1 Arg399Gln polymorphism, comprising 1,003 cases and 1,093 controls. Meanwhile, four other studies investigated the hOGG1 Ser326Cys single nucleotide polymorphism (SNP), involving 378 cases and 452 controls. The general characteristics of the included studies are presented in Table 1. The period of publication for these studies ranged from 2011 to 2016. The studies spanned populations of Caucasians and Asians, and all case groups consisted of pathologically diagnosed patients with EC. Each included study underwent Hardy–Weinberg equilibrium (HWE) examination for the genotype distribution in control groups. We utilized the chi-square test from the goodness-of-fit test to determine the HWE. Studies with *P* > 0.05 were considered to have maintained genetic balance, indicating that the data originated from the same Mendelian population. One study [27] investigating hOGG1 Ser326Cys did not meet the HWE, and thus, was excluded. The remaining studies met the criteria and were included in the analysis.

**Table 1:** Characteristics of studies included in the meta-analysis

Study author	Publication year	Country	Sample size (cases/controls)	Ethnicity	Polymorphic loci	H–W equilibrium *P*-value
Chen	2016	China	108/110	Asian	XRCC1-Arg399Gln	>0.05
Hosono	2013	Japan	91/261	Asian	XRCC1-Arg399Gln, hOGG1-Ser326Cys*	>0.05
						<0.05
Cincin	2012	Turkey	104/158	Caucasian	XRCC1-Arg399Gln, hOGG1-Ser326Cys	>0.05
Sobczuk	2012	Poland	94/114	Caucasian	XRCC1-Arg399Gln, hOGG1-Ser326Cys	>0.05
Makowska	2011	Poland	150/150	Caucasian	XRCC1-Arg399Gln, hOGG1-Ser326Cys	>0.05
Renata	2011	Poland	30/30	Caucasian	hOGG1-Ser326Cys	>0.05
Samulak	2011	Poland	456/300	Caucasian	XRCC1-Arg399Gln	>0.05

Note: Hosono’s study on hOGG1 – Ser326Cys* did not meet Hardy-Weinberg genetic equilibrium and was therefore not included in the final meta-analysis.

### 3.3 Results of quality assessment

The NOS was utilized to evaluate the methodological quality of each study. Overall, the results indicate that a single study received a score of 7 points, while three studies obtained a score of 8 points, and another three studies achieved a score of 9 points. Blinding was not implemented in any of the studies, and there was a lack of indication of allocation concealment. There were no apparent funding biases observed in any of the studies. No studies were found to have incomplete outcome data, early stoppage bias, or baseline imbalances. Table 2 provides a summary of the potential risks of bias and their corresponding ratios.

**Table 2:** Quality assessment according to NOS of each cohort study

Study	Selection				Comparability	Outcome			Total score
	Representativeness of the exposed cohort	Selection of the non-exposed cohort	Ascertainment of exposure	Demonstration that outcome	Comparability of cohorts	Assessment of outcome	Was follow-up long enough	Adequacy of follow-up of cohorts	
Chen	★	★	★	★	★★	★	★	★	9
Hosono		★	★	★	★★	★	★	★	8
Cincin	★	★	★	★	★★	★	★	★	9
Sobczuk	★	★	★	★	★★	★		★	8
Makowska	★		★	★	★★		★	★	7
Renata	★	★	★	★	★	★	★	★	8
Samulak	★	★	★	★	★★	★	★	★	9

NOS: Newcastle-Ottawa Scale.

### 3.4 Results of meta-analysis

In the meta-analysis, we assessed the association between the XRCC1-Arg399Gln SNP and susceptibility to EC. The global quantitative analysis revealed a significant relationship, with the dominant model exhibiting an OR of 1.14 (95%: 1.01–1.29), and the homozygous model yielding an OR of 1.59 (95% CI: 1.12–2.25, *P* = 0.048). Furthermore, comparison of the 399Gln allele to the 399Arg allele revealed a combined OR of 1.26 (95% CI: 1.05–1.51) (Figures 2–4).

**Figure 2:** Association between XRCC1-Arg399Gln polymorphism and EC in the overall population (Dominant genetic model).

**Figure 3:** Association between XRCC1-Arg399Gln polymorphism and EC in the overall population (Homozygous genetic model).

**Figure 4:** Association between XRCC1-Arg399Gln polymorphism and EC in the overall population (Allelic genetic model).

Given the high heterogeneity observed in the overall pooled analysis, we decided to perform subgroup analyses based on ethnicity. This was motivated by our hypothesis that differences in ethnicity could account for the observed high heterogeneity in the overall OR. Analysis of Caucasian individuals showed the dominant model OR to be 1.14 (95% CI: 1.07–1.21) and the homozygous model OR to be 1.60 (95% CI: 1.20–2.13; Figures 5 and 6). Importantly, no significant heterogeneity was detected in this population, bolstering our hypothesis that differences in ethnicity could be a contributing factor to the observed heterogeneity in the overall OR values. In the subgroup analysis of Asian individuals, however, only two studies were included. Due to the high heterogeneity and limited number of studies, we refrained from providing a detailed interpretation. The results of this subgroup analysis are presented in Table 3.

**Figure 5:** Association between XRCC1-Arg399Gln polymorphism and EC in the Caucasian population (Dominant genetic model).

**Figure 6:** Association between XRCC1-Arg399Gln polymorphism and EC in the Caucasian population (Homozygous genetic model).

**Table 3:** Analysis of the association between XRCC1 Arg399Gln polymorphism and susceptibility to endometrial cancer

Ethnic group		Genetic model	OR	95% CI	*P* value	Meta-analysis model
Overall		Allele model (Gln vs Arg)	1.26	1.05–1.51	0.001	Random effects
		Dominant model (Gln/Gln + Arg/Gln vs Arg/Arg)	1.14	1.01–1.29	0.013	Random effects
		Recessive model (Gln/Gln vs Arg/Gln + Arg/Arg)	2.02	0.96–4.26	0.06	Fixed effects
		Homozygous model (Gln/Gln vs Arg/Arg)	1.59	1.12–2.25	0.048	Random effects
		Heterozygous model (Arg/Gln vs Arg/Arg)	1.12	0.75–1.66	0.58	Fixed effects
Caucasians		Allele model (Gln vs Arg)	1.87	1.30–2.68	0.0007	Random effects
		Dominant model (Gln/Gln + Arg/Gln vs Arg/Arg)	1.14	1.07–1.21	0.490	Fixed effects
		Recessive model (Gln/Gln vs Arg/Gln + Arg/Arg)	2.77	1.25–6.11	0.01	Random effects
		Homozygous model (Gln/Gln vs Arg/Arg)	1.60	1.20–2.13	0.160	Fixed effects
		Heterozygous model (Arg/Gln vs Arg/Arg)	1.11	0.66–1.86	0.7	Fixed effects

We further examined the hOGG1-Ser326Cys polymorphism in the context of EC susceptibility. This SNP was assessed in four studies that included Caucasian individuals. Here, we found a correlation between the SNP and susceptibility to EC, with a heterozygote model OR of 1.29 (95% CI: 1.02–1.63) and an allele OR of 1.31 (95% CI: 1.07–1.60). The heterogeneity among these studies was small, prompting us to apply a fixed-effects model (Figures 7 and 8). These results underscore the importance of considering genetic variants and ethnicity in studying EC susceptibility.

**Figure 7:** Association between hOGG1-Ser326Cys polymorphism and EC in the Caucasian population (Heterozygous model).

**Figure 8:** Association between hOGG1-Ser326Cys polymorphism and EC in the Caucasian population (Allelic model).

### 3.5 Sensitivity analysis

To evaluate the potential influence of individual studies on the overall meta-analysis results, a sensitivity analysis was performed. This involved excluding one study at a time and reassessing the overall effects. The results from this analysis indicated no significant alteration in the meta-analysis outcomes upon the removal of any particular study. This confirms the robustness of our findings and suggests that our conclusions are not reliant on any single included study. However, an exception was observed in the case of the XRCC1 Arg399Gln dominant gene model. When we excluded the study by Hosono et al., which focused on Asian populations, the heterogeneity vanished, with *I* ^2^ changing from *I* ^2^ = 72.8%, *P* = 0.013 to *I* ^2^ = 0%, *P* = 0.91. This implies that the Hosono et al. study may be a significant source of heterogeneity within the dominant gene model analysis for the XRCC1 Arg399Gln polymorphism. This sensitivity analysis underscores the importance of being cautious when generalizing findings across diverse ethnic groups. Differences in genetic background and environmental exposures between populations can contribute to varying levels of heterogeneity in genetic association studies.

### 3.6 Publication bias

The funnel plots generated from the observed study exhibited symmetry, and no statistically significant evidence of publication bias was identified in the corresponding funnel plots (Figure 9). The Egger’s linear regression test was conducted to assess the presence of publication bias in the meta-analyses across various variables. The results indicated that no significant publication bias was observed (*P* > 0.05 for all), thereby providing additional support for the reliability and validity of the meta-analysis outcomes.

**Figure 9:** Funnel plot for publication bias in all included studies.

## 4 Discussion

In this comprehensive meta-analysis, we have illuminated significant associations between XRCC1-Arg399Gln and hOGG1-Ser326Cys polymorphisms and the risk of EC, particularly highlighting the influence of ethnicity on genetic susceptibility. Our findings extend the current understanding of EC etiology by demonstrating that these polymorphisms significantly elevate the risk in Caucasian populations. This emphasizes the critical role of DNA repair mechanisms in the pathogenesis of this malignancy and underscores the genetic diversity influencing disease susceptibility. Notably, the observed heterogeneity in the overall pooled analysis, which was substantially reduced in subgroup analyses based on ethnicity, provides a novel insight into the complex interplay between genetic and environmental factors in EC. These results underscore the need for personalized approaches in both risk assessment and therapeutic strategies, considering the genetic background of individual patients. Furthermore, the rigorous methodological approach adopted in this study, adhering to the PRISMA guidelines and employing the NOS for quality assessment, ensures the robustness and reliability of our findings. This study, therefore, contributes substantially to the field by providing a more nuanced understanding of the genetic factors in EC and sets the stage for future research to explore other DNA repair gene polymorphisms across diverse ethnicities.

DNA is the repository of genetic information, and its integrity is pivotal to cell survival and function. However, DNA can be compromised by various endogenous and exogenous factors leading to DNA damage [30–33]. The human body has evolved a system of DNA repair mechanisms that ensure the stability and fidelity of DNA [34]. These mechanisms include photorepair, mismatch repair, single and double-strand break repair, BER, and nucleotide excision repair [35,36]. The role of these DNA repair systems is crucial in maintaining genomic integrity and any malfunction, often due to mutations in the DNA repair genes, could result in carcinogenesis [37–39]. Polymorphisms in DNA repair genes have been implicated in the pathogenesis of several malignancies. SNPs in XRCC1 and hOGG1, two key genes in the BER pathway, have been linked to an elevated risk of various malignancies [40–43]. Yet, the association between these polymorphisms and EC risk remains inconclusive. Our study aimed to elucidate the potential association between XRCC1 Arg399Gln and hOGG1 Ser326Cys SNPs and EC risk.

Our meta-analysis incorporated seven case–control studies, encompassing 1,033 cases and 1,123 controls. We observed a significantly increased risk of EC associated with the XRCC1 Arg399Gln polymorphism. The 399Gln allele was associated with an increased risk of EC compared with the 399Arg allele (OR = 1.26, 95% CI: 1.05–1.51). Specifically, carriers of the Gln/Gln genotype were at significantly higher risk compared to those carrying the Arg/Arg genotype (OR = 1.59, 95% CI: 1.12–2.25). These findings indicate that the XRCC1 Arg399Gln polymorphism is a potential susceptibility factor for EC, particularly in those carrying the Gln/Gln genotype. Subgroup analysis based on ethnicity demonstrated similar results in the Caucasian population and showed reduced inter-study heterogeneity, suggesting that the XRCC1 Arg399Gln polymorphism could be a significant risk factor, particularly among Caucasian females. However, due to the limited number of studies available, we refrained from providing detailed interpretation for the Asian population subgroup. We further explored the association of the hOGG1 Ser326Cys polymorphism with EC susceptibility. All studies assessing this SNP included Caucasian populations. This SNP was also associated with an increased risk of EC, with the 326Cys allele potentially increasing the risk of EC in Caucasians. Notably, inter-study heterogeneity was reduced in the ethnic-specific subgroups, suggesting that the overall heterogeneity mainly originates from the variations in ethnic background. Furthermore, the sensitivity analysis showed that the overall results were robust and not significantly influenced by any single study.

The critical roles of XRCC1 and hOGG1 polymorphisms in DNA repair and their impact on EC development offer transformative potential for early detection and prevention strategies. Enhanced screening and preventive measures for individuals with these genotypes could significantly reduce carcinoma risk. Such genetic insights pave the way for personalized treatments, considering these polymorphisms considerably affect therapeutic responses [44]. Furthermore, the intricate interplay of gene–gene and gene–environment interactions, particularly involving XRCC1 and hOGG1, might modulate EC susceptibility [45]. Integrating genetic markers like XRCC1-Arg399Gln and hOGG1-Ser326Cys into routine screening, especially in populations with a high genetic predisposition, could improve early detection and prognosis [46]. However, challenges in early EC detection persist, marked by rising incidence and mortality rates, and the lack of effective screening tests [47,48]. The gap in early diagnostic methods, underscored by the absence of comprehensive screening programs and reliable biomarkers, calls for urgent research in this area. Advances in categorizing EC through The Cancer Genome Atlas into distinct molecular groups provide a more objective framework for prognosis and treatment [49]. While most EC cases are effectively managed through surgery in early stages, advanced stages pose treatment challenges, with current options being largely palliative. Emerging targeted therapies, especially those focusing on DNA repair mechanisms and tailored to specific genomic alterations like microsatellite instability and ARID1A mutations, show promise, particularly with the use of PARP and ATR inhibitors [50]. Our comprehensive review highlights the imperative of integrating genetic risk assessment into routine EC management and developing robust early detection methods and novel targeted therapies, an approach vital for enhancing patient outcomes and quality of life in EC.

Our meta-analysis underscores the pivotal role of genetic polymorphisms in EC susceptibility, emphasizing the influence of genetic variants and ethnicity. Despite using funnel plots and Egger’s regression to mitigate publication bias, a key strength of our study, limitations persist. These include a limited number of studies focused primarily on Caucasian and Asian populations, constraining broader applicability. Additionally, the exclusion of studies not adhering to HWE may have omitted valuable data, as deviations can occur due to natural selection or smaller sample sizes. Incorporating such studies in future sensitivity analyses could enhance the comprehensiveness and interpretation of findings, further informing individualized prevention strategies for EC.

## 5 Conclusions

In conclusion, our systematic review and meta-analysis suggest that XRCC1-Arg399Gln and hOGG1-Ser326Cys polymorphisms may be associated with an increased risk of EC, especially in Caucasian women. These findings underscore the importance of genetic factors in the etiology of EC, highlighting the potential role of DNA repair mechanisms in disease susceptibility. Further comprehensive and well-designed studies are warranted to confirm these findings in diverse ethnic groups.

## References

[1] Cripe J, Handorf E, Brown J, Jain A, Rubin S, Mantia-Smaldone G. National cancer database report of lymphadenectomy trends in endometrial cancer. Int J Gynecol Cancer. 2017;27(7):1408–15.10.1097/IGC.000000000000100528525495

[2] Huvila J, Pors J, Thompson EF, Gilks CB. Endometrial carcinoma: molecular subtypes, precursors and the role of pathology in early diagnosis. J Pathol. 2021;253(4):355–65.10.1002/path.560833368243

[3] Miller KD, Nogueira L, Devasia T, Mariotto AB, Yabroff KR, Jemal A, et al. Cancer treatment and survivorship statistics, 2022. CA Cancer J Clin. 2022;72(5):409–36.10.3322/caac.2173135736631

[4] Ren X, Liang J, Zhang Y, Jiang N, Xu Y, Qiu M, et al. Single-cell transcriptomic analysis highlights origin and pathological process of human endometrioid endometrial carcinoma. Nat Commun. 2022;13(1):6300.10.1038/s41467-022-33982-7PMC958807136273006

[5] Gao S, Zhao T, Meng F, Luo Y, Li Y, Wang Y. Circular RNAs in endometrial carcinoma (Review). Oncol Rep. 2022;48(6):212.10.3892/or.2022.8427PMC960825636263622

[6] Semaan A, Ali-Fehmi R, Munkarah AR, Bandyopadhyay S, Morris RT, Rizk S, et al. Clinical/pathologic features and patient outcome in early onset endometrial carcinoma: a population based analysis and an institutional perspective from the Detroit metropolitan area, Michigan. Gynecol Oncol. 2012;124(2):265–9.10.1016/j.ygyno.2011.09.02722044605

[7] Aune D, Sen A, Vatten LJ. Hypertension and the risk of endometrial cancer: a systematic review and meta-analysis of case–control and cohort studies. Sci Rep. 2017;7:44808.10.1038/srep44808PMC538428028387226

[8] Wu QJ, Li YY, Tu C, Zhu J, Qian KQ, Feng TB, et al. Parity and endometrial cancer risk: a meta-analysis of epidemiological studies. Sci Rep. 2015;5:14243.10.1038/srep14243PMC464270526373341

[9] Bogani G, Ray-Coquard I, Concin N, Ngoi NYL, Morice P, Enomoto T, et al. Clear cell carcinoma of the endometrium. Gynecol Oncol. 2022;164(3):658–66.10.1016/j.ygyno.2022.01.01235063279

[10] Liang X, Zeng H, Chen S, Jiang M, Liu S, Fan J. Ovarian metastasis risk factors in endometrial carcinoma: a systematic review and meta-analysis. Eur J Obstet Gynecol Reprod Biol. 2021;267:245–55.10.1016/j.ejogrb.2021.11.01634837854

[11] Garg V, Jayaraj AS, Kumar L. Novel approaches for treatment of endometrial carcinoma. Curr Probl Cancer. 2022;46(5):100895.10.1016/j.currproblcancer.2022.10089535986972

[12] Gladyshev VN, Kritchevsky SB, Clarke SG, Cuervo AM, Fiehn O, de Magalhães JP, et al. Molecular damage in aging. Nat Aging. 2021;1(12):1096–106.10.1038/s43587-021-00150-3PMC995751636846190

[13] van den Heuvel D, van der Weegen Y, Boer DEC, Ogi T, Luijsterburg MS. Transcription-coupled DNA repair: from mechanism to human disorder. Trends Cell Biol. 2021;31(5):359–71.10.1016/j.tcb.2021.02.00733685798

[14] Oh JM, Myung K. Crosstalk between different DNA repair pathways for DNA double strand break repairs. Mutat Res Genet Toxicol Environ Mutagen. 2022;873:503438.10.1016/j.mrgentox.2021.50343835094810

[15] Baxter JS, Zatreanu D, Pettitt SJ, Lord CJ. Resistance to DNA repair inhibitors in cancer. Mol Oncol. 2022;16(21):3811–27.10.1002/1878-0261.13224PMC962778335567571

[16] Stead ER, Bjedov I. Balancing DNA repair to prevent ageing and cancer. Exp Cell Res. 2021;405(2):112679.10.1016/j.yexcr.2021.112679PMC836178034102225

[17] Bhardwaj A, Bahl C, Sharma S, Singh N, Behera D. Interactive potential of genetic polymorphism in Xenobiotic metabolising and DNA repair genes for predicting lung cancer predisposition and overall survival in North Indians. Mutat Res Genet Toxicol Environ Mutagen. 2018;826:15–24.10.1016/j.mrgentox.2017.12.00629412865

[18] Romanowicz-Makowska H, Smolarz B, Houli A, Szyłło K. Single polymorphism in DNA base excision repair genes XRCC1 and hOGG1 and the risk of endometrial carcinoma in the Polish population. Pol J Pathol. 2011;62(2):89–94.21866464

[19] Zhang XQ, Li L. A meta-analysis of XRCC1 single nucleotide polymorphism and susceptibility to gynecological malignancies. Medicine (Baltimore). 2021;100(50):e28030.10.1097/MD.0000000000028030PMC867795334918657

[20] Romanowicz-Makowska H, Smolarz B, Houli A, Szyłło K. Single nucleotide polymorphism in DNA base excision repair genes XRCC1 and hOGG1 and the risk of endometrial carcinoma in the Polish population. Pol J Pathol: Off J Pol Soc Pathol. 2011;62(2):89–94.21866464

[21] Shi Y, Xu W, Zhang X. Association of the hOGG1 Ser326Cys polymorphism with gynecologic cancer susceptibility: a meta-analysis. Biosci Rep. 2020;40(12). 10.1042/BSR20203245 PMC769319733210702

[22] Krupa R, Sobczuk A, Popławski T, Wozniak K, Blasiak J. DNA damage and repair in endometrial cancer in correlation with the hOGG1 and RAD51 genes polymorphism. Mol Biol Rep. 2011;38(2):1163–70.10.1007/s11033-010-0214-zPMC302451520602259

[23] Page MJ, McKenzie JE, Bossuyt PM, Boutron I, Hoffmann TC, Mulrow CD, et al. The PRISMA 2020 statement: an updated guideline for reporting systematic reviews. BMJ. 2021;372:n71.10.1136/bmj.n71PMC800592433782057

[24] Wells G, editor. The Newcastle-Ottawa Scale (NOS) for assessing the quality of non-randomised studies in meta-analyses. Symposium on systematic reviews: Beyond the basics; 2014.

[25] Chen L, Liu MM, Liu H, Lu D, Zhao XD, Yang XJ. ERCC1 and XRCC1 but not XPA single nucleotide polymorphisms correlate with response to chemotherapy in endometrial carcinoma. Onco Targets Ther. 2016;9:7019–28.10.2147/OTT.S110976PMC511787727895494

[26] Cincin ZB, Iyibozkurt AC, Kuran SB, Cakmakoglu B. DNA repair gene variants in endometrial carcinoma. Med Oncol. 2012;29(4):2949–54.10.1007/s12032-012-0162-722271435

[27] Hosono S, Matsuo K, Ito H, Oze I, Hirose K, Watanabe M, et al. Polymorphisms in base excision repair genes are associated with endometrial cancer risk among postmenopausal Japanese women. Int J Gynecol Cancer. 2013;23(9):1561–8.10.1097/IGC.0b013e3182a80a7e24172093

[28] Samulak D, Romanowicz-Makowska H, Smolarz B, Kulig A, Sporny S. Association between Arg399Gln polymorphism of X-ray repair cross-complementing 1 (XRCC1) gene and sporadic endometrial cancer in the Polish population. Eur J Gynaecol Oncol. 2011;32(5):491–5.22053659

[29] Sobczuk A, Poplawski T, Blasiak J. Polymorphisms of DNA repair genes in endometrial cancer. Pathol Oncol Res. 2012;18(4):1015–20.10.1007/s12253-012-9537-5PMC344805022544315

[30] Attar R, Cacina C, Sozen S, Attar E, Agachan B. DNA repair genes in endometriosis. Genet Mol Res. 2010;9(2):629–36.10.4238/vol9-2gmr77920391347

[31] Ricceri F, Matullo G, Vineis P. Is there evidence of involvement of DNA repair polymorphisms in human cancer? Mutat Res. 2012;736(1–2):117–21.10.1016/j.mrfmmm.2011.07.01321864546

[32] Matthews HK, Bertoli C, de Bruin RAM. Cell cycle control in cancer. Nat Rev Mol Cell Biol. 2022;23(1):74–88.10.1038/s41580-021-00404-334508254

[33] Clay DE, Fox DT. DNA damage responses during the cell cycle: insights from model organisms and beyond. Genes (Basel). 2021;12(12). 10.3390/genes12121882 PMC870101434946831

[34] Zhao S, Tadesse S, Kidane D. Significance of base excision repair to human health. Int Rev Cell Mol Biol. 2021;364:163–93.10.1016/bs.ircmb.2021.05.00234507783

[35] Qian B, Zhang H, Zhang L, Zhou X, Yu H, Chen K. Association of genetic polymorphisms in DNA repair pathway genes with non-small cell lung cancer risk. Lung Cancer. 2011;73(2):138–46.10.1016/j.lungcan.2010.11.01821195504

[36] Demin AA, Hirota K, Tsuda M, Adamowicz M, Hailstone R, Brazina J, et al. XRCC1 prevents toxic PARP1 trapping during DNA base excision repair. Mol Cell. 2021;81(14):3018–30.e5.10.1016/j.molcel.2021.05.009PMC829432934102106

[37] Goode EL, Ulrich CM, Potter JD. Polymorphisms in DNA repair genes and associations with cancer risk. Cancer Epidemiol Biomarkers Prev. 2002;11(12):1513–30.12496039

[38] Dimberg J, Skarstedt M, Slind Olsen R, Andersson RE, Matussek A. Gene polymorphism in DNA repair genes XRCC1 and XRCC6 and association with colorectal cancer in Swedish patients. Apmis. 2016;124(9):736–40.10.1111/apm.1256327328741

[39] Allkanjari K, Baldock RA. Beyond base excision repair: an evolving picture of mitochondrial DNA repair. Biosci Rep. 2021;41(10):BSR20211320.10.1042/BSR20211320PMC852720734608928

[40] Sanjari Moghaddam A, Nazarzadeh M, Bidel Z, Karamatinia A, Darvish H, Mosavi Jarrahi A. hOGG1 gene polymorphism and breast cancer risk: a systematic review and meta-analysis study. Breast J. 2018;24(1):70–3.10.1111/tbj.1284228608470

[41] Guo CL, Han FF, Wang HY, Wang L. Meta-analysis of the association between hOGG1 Ser326Cys polymorphism and risk of colorectal cancer based on case–control studies. J Cancer Res Clin Oncol. 2012;138(9):1443–8.10.1007/s00432-012-1197-zPMC1182416222526153

[42] Bahreini F, Rayzan E, Rezaei N. microRNA-related single-nucleotide polymorphisms and breast cancer. J Cell Physiol. 2021;236(3):1593–605.10.1002/jcp.2996632716070

[43] Donda KT, Torres BA, Khashu M, Maheshwari A. Single nucleotide polymorphisms in neonatal necrotizing enterocolitis. Curr Pediatr Rev. 2022;18(3):197–209.10.2174/157339631866622011709162135040407

[44] Chow RD, Michaels T, Bellone S, Hartwich TMP, Bonazzoli E, Iwasaki A, et al. Distinct mechanisms of mismatch-repair deficiency delineate two modes of response to anti-PD-1 immunotherapy in endometrial carcinoma. Cancer Discov. 2023;13(2):312–31.10.1158/2159-8290.CD-22-0686PMC990526536301137

[45] Peng Q, Lu Y, Lao X, Chen Z, Li R, Sui J, et al. Association between OGG1 Ser326Cys and APEX1 Asp148Glu polymorphisms and breast cancer risk: a meta-analysis. Diagn Pathol. 2014;9:108.10.1186/1746-1596-9-108PMC406481124893568

[46] Bianco B, Barbosa CP, Trevisan CM, Laganà AS, Montagna E. Endometrial cancer: a genetic point of view. Transl Cancer Res. 2020;9(12):7706–15.10.21037/tcr-20-2334PMC879794435117373

[47] Smolarz B, Michalska MM, Samulak D, Wojcik L, Romanowicz H. Studies of correlations between single nucleotide polymorphisms of DNA repair genes and endometrial cancer in polish women. Anticancer Res. 2018;38(9):5223–9.10.21873/anticanres.1284630194171

[48] Sznurkowski JJ, Knapp P, Bodnar L, Bidziński M, Jach R, Misiek M, et al. Recommendations of the polish gynecological oncology society for the diagnosis andtreatment of endometrial cancer. Curr Gynecol Oncol. 2017;15(1):34–44.

[49] Kuhn TM, Dhanani S, Ahmad S. An overview of endometrial cancer with novel therapeutic strategies. Curr Oncol. 2023;30(9):7904–19.10.3390/curroncol30090574PMC1052834737754489

[50] MacKay HJ, Freixinos VR, Fleming GF. Therapeutic targets and opportunities in endometrial cancer: update on endocrine therapy and nonimmunotherapy targeted options. Am Soc Clin Oncol Educ Book. 2020;40:1–11.10.1200/EDBK_28049532239967

